# Cognitive dysfunction associated with COVID-19: Prognostic role of circulating biomarkers and microRNAs

**DOI:** 10.3389/fnagi.2022.1020092

**Published:** 2022-10-04

**Authors:** Marissa Alvarez, Erick Trent, Bruno De Souza Goncalves, Duane G. Pereira, Raghav Puri, Nicolas Anthony Frazier, Komal Sodhi, Sneha S. Pillai

**Affiliations:** Department of Surgery, Biomedical Sciences and Medicine, Joan C. Edwards School of Medicine, Marshall University, Huntington, WV, United States

**Keywords:** COVID-19, cognitive impairment, neurodegenerative diseases, circulating biomarkers, microRNAs

## Abstract

COVID-19 is renowned as a multi-organ disease having subacute and long-term effects with a broad spectrum of clinical manifestations. The evolving scientific and clinical evidence demonstrates that the frequency of cognitive impairment after COVID-19 is high and it is crucial to explore more clinical research and implement proper diagnostic and treatment strategies. Several central nervous system complications have been reported as comorbidities of COVID-19. The changes in cognitive function associated with neurodegenerative diseases develop slowly over time and are only diagnosed at an already advanced stage of molecular pathology. Hence, understanding the common links between COVID-19 and neurodegenerative diseases will broaden our knowledge and help in strategizing prognostic and therapeutic approaches. The present review focuses on the diverse neurodegenerative changes associated with COVID-19 and will highlight the importance of major circulating biomarkers and microRNAs (miRNAs) associated with the disease progression and severity. The literature analysis showed that major proteins associated with central nervous system function, such as Glial fibrillary acidic protein, neurofilament light chain, p-tau 181, Ubiquitin C-terminal hydrolase L1, S100 calcium-binding protein B, Neuron-specific enolase and various inflammatory cytokines, were significantly altered in COVID-19 patients. Furthermore, among various miRNAs that are having pivotal roles in various neurodegenerative diseases, miR-146a, miR-155, Let-7b, miR-31, miR-16 and miR-21 have shown significant dysregulation in COVID-19 patients. Thus the review consolidates the important findings from the numerous studies to unravel the underlying mechanism of neurological sequelae in COVID-19 and the possible association of circulatory biomarkers, which may serve as prognostic predictors and therapeutic targets in future research.

## Introduction

Coronavirus disease 2019 (COVID-19), the disease caused by severe acute respiratory syndrome coronavirus 2 (SARS-CoV-2), has created morbidity and mortality at an unprecedented scale globally and was declared a pandemic by the World Health Organization (WHO) in March 2020 (Nalbandian et al., 2021). It was initially detected in Wuhan, China, which triggered a severe acute respiratory syndrome, contaminating more than 175 million people after one year and leading to the death of 3.8 million people worldwide (Huang et al., 2020; Hui et al., 2020; Wu et al., 2020a; Lopez-Leon et al., 2021). SARS-CoV-2 is a betacoronavirus, a member of the subfamily *Coronavirinae*, having a single-stranded positive-sense RNA genome (Wang et al., 2020b). SARS-CoV-2 is made up of at least 29 proteins, four of which are structural proteins, and the others are non-structural proteins (Yao et al., 2020). SARS-CoV-2 is prone to genetic evolution through mutations over time in human hosts. This leads to the generation of mutant variants having diverse characteristics than their ancestral strains. Several variants of SARS-CoV-2 have been described during the course of this pandemic and WHO has classified them based on their impact on public health. Currently, there are five SARS-CoV-2 variants of concern (VOC), Alpha, Beta, Gamma, Delta, and Omicron, and two SARS-CoV-2 variants of interest (VOI), Lambda and Mu (WHO SARS-CoV-2 Variants) (Liu et al., 2022). The emergence of these new SARS-CoV-2 variants are posing threats to vaccine development and other therapeutic options.

Several scientific and clinical studies have shown that subacute and long-term effects of COVID-19 can affect multiple organ systems (Gupta et al., 2020a). It is reported that the mechanism of infection and replication of SARS-CoV-2 is similar to that of SARS-CoV and MERS-CoV. The angiotensin-converting enzyme-2 (ACE-2) receptors are the primary binding receptors for the viral particle and are found highly expressed in alveolar epithelial cells of lungs, vascular endothelial cells, and enterocytes but can also be found in other organs, such as kidney, liver, and gastrointestinal tract (Azer, 2020; Bhavana et al., 2020; Harrison et al., 2020; Parasher, 2021). The internalization of the virus in host cells results in different inflammatory changes such as edema, necrosis, and tissue dysfunction. These changes can cause a cytokine storm, promoting changes in the immune response that cause excessive damage to the lung, gastrointestinal, neurological, and cardiopulmonary systems (Azer, 2020; Bhavana et al., 2020; Harrison et al., 2020; Rizzo et al., 2020; Xu et al., 2020; Anka et al., 2021).

As SARS-CoV-2 has the ability to affect different organs, recent clinical studies have demonstrated that there is an increased risk of long-term health problems in patients who have survived infection with SARS-CoV-2 (Seyedalinaghi et al., 2021). The most recurrent long-term complication is respiratory problems that may further develop pulmonary fibrosis, arterial complications, venous thrombo-embolic late complications associated with a hyperinflammatory and hypercoagulable state (Lodigiani et al., 2020; Puntmann et al., 2020). Likewise, cardiac dysfunction can be caused due to structural damage to the myocardium, pericardium, and conduction system, triggering arrhythmias in a large proportion of patients (Lindner et al., 2020; Liu et al., 2020). Renal lesions have also been reported in approximately 20-31% of patients who developed the severe form of COVID-19. The reduced glomerular filtration was related to extensive acute tubular necrosis observed in renal biopsies (Kudose et al., 2020). Diabetic ketoacidosis, liver dysfunction, joint pain, muscle weekness and dermatologic manifestations were also observed in post-covid patients (Freeman et al., 2020; Suwanwongse and Shabarek, 2021). In addition, late complications are reported in the central and peripheral nervous system, promoting decreased awareness and absorption, difficulties with concentration, disturbed memory, difficulty in communication, anxiety, depression, sleep problems, and olfactory and taste losses (Paybast et al., 2020; Varatharaj et al., 2020; Huang et al., 2021a). Figure 1 demonstrates the various complications associated with COVID-19.

**FIGURE 1:** Schematic representation showing the potential complications of COVID-19 causing wide range of complications in various organ systems.

The present review aims to elucidate the underlying mechanism that links COVID-19 with neurodegenerative changes that lead to cognitive dysfunction. As patients infected with SARS-CoV-2 are stratified according to their clinical manifestations, such as symptoms, oxygen saturation, and blood pressure (Malik et al., 2021), these manifestations are apparent at the late stages of infection, especially for neurological complications. Identifying factors that can lead to complications during the disease early is extremely important since it can significantly influence the quality of care and adequate treatment. It would be valuable to reveal the alterations of plasma biomarkers in various cognitive impairment stages since the cognitive manifestations are one of the most concerned post covid complications. Hence, based on recent literature, we will provide clinicians with updated and practical information on the role of circulating biomarkers and miRNAs in COVID-19-associated cognitive dysfunction that may act as possible therapeutic targets and prognostic predictors in future studies.

## Materials and methods

The purpose of this review is to highlight the importance of cognitive dysfunction and neurodegenerative changes associated with COVID-19 and the dysregulation of circulating biomarkers and miRNAs in the clinical condition being studied. A systematic search of relevant research articles was performed using the databases, namely, PubMed, ProQuest, Science Direct, and Google Scholar. The electronic search was conducted using a combination of search terms related to the following keywords: “COVID-19” OR “SARS-CoV-2” OR “Post COVID-19 complications” OR “Cognitive dysfunction” OR “Neurodegeneration” OR “Circulating Biomarkers” OR “miRNAs”. The articles retrieved from our search were further distinguished for relevancy. The inclusion and exclusion criteria were set to only evaluate articles published from 2000 to 2022 in order to limit this search. Moreover, articles that contain only abstracts without their full text and published in languages other than English were excluded.

## COVID-19-associated cognitive dysfunction and neurodegeneration

### COVID-19-associated cognitive dysfunction

As the population of patients recovering from COVID-19 grows, it is important to establish an understanding of the multi-organ dysfunction associated with post- COVID-19 complications. Of note, neurological manifestations in COVID-19 patients have been reported, showing a close correlation between COVID-19 and future development of neurodegenerative diseases (Wu et al., 2020b; Taquet et al., 2021; Frontera et al., 2022; Li et al., 2022a). It has also been established that the likelihood of developing COVID-19-associated cognitive impairment and the severity of these deficits is associated with the severity of the SARS-CoV-2 infection and the subsequent increases in specific circulating inflammatory mediators and biomarkers (Becker et al., 2021; Miskowiak et al., 2021; Zeng et al., 2022). Alternatively, some studies have demonstrated that even non-hospitalized COVID-19 patients have developed cognitive-associated post-COVID-19 symptoms, suggesting that regardless of illness severity, cognitive dysfunction can arise (Graham et al., 2021; Hadad et al., 2022; Van Kessel et al., 2022). Report shows that COVID-19-associated cognitive impairment can arise during post-acute COVID-19 infection 3 weeks following diagnosis, and 31.2% of participants experience cognitive dysfunction within the first week of symptoms (Davis et al., 2021). Another study found that 22% of individuals infected with SARS-CoV-2 developed symptoms of cognitive impairment, which remained after 12 weeks following their diagnosis (Ceban et al., 2022). These deficits can last for a prolonged period of time and clinically relevant cognitive impairments in verbal learning and executive function were found in 48% of patients 1 year following the onset of symptoms (Miskowiak et al., 2022).

Likewise, another report identified abnormalities in executive function, attention, and phonemic fluency in post-COVID-19 patients (Hadad et al., 2022). The results of a systemic review showed a high frequency of cognitive impairment after COVID-19 infection with defects in processing speed, inattention, or executive dysfunction (Tavares-Junior et al., 2022). A post-COVID-19 community clinic compared Montreal Cognitive Assessment (MoCA) index scores of participants who reported cognitive symptoms and found that index scores were significantly worse in language, executive function, and attention (Crivelli et al., 2022). With increasing severity of infection with SARS-CoV-2, there are corresponding increases in both the likelihood of developing cognitive dysfunction as well as the severity of the cognitive dysfunction in those who develop these sequelae (Wang et al., 2021). For these reasons, it is imperative to understand the underlying mechanisms by which covid-associated cognitive dysfunction and neurodegeneration occur.

### COVID-19-associated neurodegeneration

The neurological complications of COVID-19 include damage to the central and the peripheral nervous system that consists of neuronal damage, neuroinflammation, rupture of the blood brain barrier, microvasculitis and hypoxia (Ellul et al., 2020; Boldrini et al., 2021). ACE2 receptors within the central nervous system (CNS) are most highly concentrated within the substantia nigra, ventricles, middle temporal gyrus, posterior cingulate cortex, olfactory bulb, motor cortex, and brainstem (Iodice et al., 2021). The disruption of the normal physiological functions of these areas due to infection with SARS-CoV-2 has been postulated to be a potential explanation for many of the reported symptoms associated with the long-Covid syndrome. This was validated by an observational study that examined cortical metabolism in the subacute and chronic (>6 months) stages of illness and found that hypometabolism in the frontoparietal and temporal cortex was associated with cognitive impairment (Hosp et al., 2021). Long- COVID-19 brain fog in patients has presented with abnormal FDG-PET scan results, with hypometabolic regions localized mostly to the anterior and posterior cingulate cortices (Hugon et al., 2022). The cingulate cortex plays a role in a variety of neurological functions including memory, emotions, and decisive action taking. The abundance of ACE2 receptors in this area could additionally provide some insight into their experience of brain fog (Hugon et al., 2022).

There are numerous potential mechanisms by which SARS-CoV-2 could access the CNS to elicit these pathologies, which can be broadly classified into direct invasion and indirect hematological entry following inflammatory mediated neurodegeneration of the blood-brain-barrier (BBB) (Iodice et al., 2021). Direct neurological invasion is hypothesized to occur through the olfactory epithelium and the cribriform plate into the olfactory bulbs following nasal inhalation of aerosolized droplets containing the infectious viral load. Additionally, it has been suggested that SARS-CoV-2 penetration into the CNS can result in heightened neuroinflammation which may cause neurodegeneration or exacerbate existing neuroinflammation from preexisting comorbidities such as Alzheimer’s dementia and Parkinson’s disease, leading to the development of neuropsychological symptoms (Iodice et al., 2021).

Hematological spread is another proposed mechanism by which SARS-CoV-2 can gain access to the CNS. One possible mechanism involves the attachment of SARS-CoV-2 to ACE2 expressed on BBB endothelial cells and the induction of neuroinflammation, which weakens the protective barrier of the brain and thus provides access for the virus. It is also hypothesized that it is possible that the virus may circumvent BBB altogether by infecting CNS-infiltrating macrophages and monocytes (Zhou et al., 2020b). Furthermore, astrocytes, a vital component of the BBB, can receive signals from circulating pro-inflammatory cytokines, generated in response to viral infection in the lungs, which in turn cause SARS-CoV-2 to enter the CNS and induce neuroinflammation (Murta et al., 2020). Moreover, SARS-CoV-2 can elicit the pro-inflammatory phenotype of microglia, the native immune cells in the CNS, which up-regulate the expression of genes involved in neuroinflammation (Amruta et al., 2021). In addition, it has been demonstrated that SARS-CoV-2 infection can facilitate neuronal injury, encephalitis, fibrosis, thrombosis and axonal damage (Bradley et al., 2020; Turski et al., 2020; Wang et al., 2020a). As, COVID-19-associated pathological changes are characterized by distinct changes in the levels of specific circulating biomarkers, the expression profile of these biomarkers may demonstrate a link between various disease states. The Schematic representation of various neurodegenerative changes associated with COVID-19 is shown in Figure 2. Understanding the changes in expression of these circulating biomarkers may provide insights into the holistic understanding of the underlying process by which COVID-19 long-haulers experience their cognitive dysfunction.

**FIGURE 2:** Schematic representation showing the neuronal infection of SARS-CoV-2 virus and CNS damage caused by the infection that leads to cognitive dysfunction and neurodegenerative diseases. Angiotensin-converting enzyme-2 (ACE-2), Alzheimer’s disease (AD), Parkinson’s disease (PD), Multiple sclerosis (MS), Amyotrophic lateral sclerosis (ALS), Multiple system atrophy (MSA), Ischemia stroke (IS).

## Role of circulating biomarkers in COVID-19-associated cognitive dysfunction

Circulating biomarkers present a promising approach in the research and clinical practice of various diseases including neurodegenerative diseases as they are minimally invasive, highly cost-effective and provide high specificity (Solfrizzi et al., 2006; Pillai et al., 2020; Lakhani et al., 2021; Kivisakk et al., 2022). The prognostic utility of plasma biomarkers in neuroinflammation, vascular injury, and cognitive dysfunction may aid in the management of clinical care and treatment strategies. Hence in this section, we are highlighting the importance of some key biomarkers of cognitive decline and neurodegeneration that are altered in COVID-19 for their future application in research on therapeutic targets and prognostic deliberations of COVID-19- associated cognitive dysfunction. A summary of the findings are illustrated in Table 1.

**TABLE 1:** Summary of circulating biomarkers associated with neurological dysfunction showing potential dysregulation in COVID-19.

Biomarker	Source	Function	Pathophysiology	Status in neurodegenerative diseases	Patients’ information	Status in COVID-19	References
GFAP	Serum/ plasma	Provides stability to astrocytes influencing their shape and movement.	Astrocytes damage and inflammation	AD- increased PD- increased MS- increased	1. 47 COVID-19 patients divided into 3 groups related to systemic disease severity. 2. 100 COVID-19 patients classified into three main groups: mild, moderate and severe patients. 3. 58 COVID-19 patients divided into 3 groups related to disease severity. 4. 251 hospitalized COVID-19 patients aged between 60-83 years without a history of dementia	Significantly increased	Eng et al., 2000; Elahi et al., 2020; Kanberg et al., 2020, 2021; Frontera et al., 2022; Heimfarth et al., 2022; Kim et al., 2022; Sahin et al., 2022
NFL	Serum/ plasma	Provide cytoskeletal stability and allow for radial growth of neurons.	Neuroaxonal injury	AD- increased PD- increased ALS- increased HD- increased LBD- increased	1. 104 COVID-19 patients 2. COVID-19 Patients classified into 3 groups according to the disease severity: mild (n = 24), moderate (n = 28), and severe (n = 48). 3. 142 hospitalized COVID-19 4. 251 hospitalized COVID-19 patients aged between 60-83 years without a history of dementia 5. 57 hospitalized Covid-19 patients without major neurological manifestations	Significantly increased	Yuan et al., 2017; Gaetani et al., 2019; Palermo et al., 2020; Rajan et al., 2020; De Lorenzo et al., 2021; Kanberg et al., 2021; Prudencio et al., 2021; Verde et al., 2021, 2022; Chouliaras et al., 2022; Frontera et al., 2022; Thijssen et al., 2022; Zanella et al., 2022
P-tau 181	Serum/ plasma	Maintaining neuronal microtubule integrity by providing stability and encouraging assembly.	Form neurofibrillary tangles	AD- increased	1. 16 COVID-19 volunteers without neurological symptoms and 8 COVID-19 volunteers with neurological symptoms 2. 251 hospitalized COVID-19 patients aged between 60-83 years without a history of dementia	Significantly increased	Metaxas and Kempf, 2016; Wang and Mandelkow, 2016; Moscoso et al., 2021; Sun et al., 2021; Frontera et al., 2022; Smirnov et al., 2022
UCH-L1	Plasma	Removing ubiquitin from their target proteins maintaining the nervous system integrity.	Changes in regulating the function of various synapses influencing their maintenance, transmission, and plasticity.	PD- increased AD-increased FA- increased	1. 27 hospitalized COVID-19 patients aged 54-76 years without major neurological manifestations 2. 251 hospitalized COVID-19 patients aged between 60-83 years without a history of dementia 3. 104 COVID-19 patients aged 49- 67	Significantly increased	Bishop et al., 2016; Zeitlberger et al., 2018; Cooper et al., 2020; Ng et al., 2020; De Lorenzo et al., 2021; Bogdan et al., 2022; Frontera et al., 2022
S100B	Serum	Regulation of cell proliferation and cytoskeletal structure	Cause astrocyte damage and injury	AD- increased PD- increased ALS- increased MS- increased	1. 74 hospitalized COVID-19 patients 2. 64 COVID-19 patients (34 mild cases; 30 severe cases) 3. 57 patients hospitalized with COVID-19 4. 58 COVID-19 Patients classified into mild (n = 17), moderate (n = 18), and severe (n = 23).	Significantly increased	Steiner et al., 2007; Lam et al., 2013; Barateiro et al., 2016; Serrano et al., 2017; Cristovao and Gomes, 2019; Aceti et al., 2020; Angelopoulou et al., 2021; Mete et al., 2021; Savarraj et al., 2021; Sahin et al., 2022
NSE	Serum/ plasma	Regulating neuronal growth, differentiation, survival.	Cause axonal injury and neuroinflammation	AD-increased HD-increased BPAN-increased	1. 252 COVID-19 patients classified into 3 groups according to the disease severity. 2. 128 hospitalized COVID-19 patients 3. 57 COVID-19 hospitalized patients	Significantly increased	Chaves et al., 2010; Ciancarelli et al., 2014; Polcyn et al., 2017; Takano et al., 2017; Haque et al., 2018; Wei et al., 2020; Cione et al., 2021; Savarraj et al., 2021
Inflammatory cytokines	Serum	Mobilization of immune cells	Cytokine storm implicated in neurotoxicity, disruption of the integrity of BBB, neuroglial cells activation, and neuroinflammation	AD-increased	1. 57 COVID-19 hospitalized patients 2. 43 COVID-19 patients with mild-moderate (*n* = 39) and severe (*n* = 14) 3. 33 COVID-19 patients 4. 60 COVID-19 patients divided in to two subgroup, clinical group (*n* = 32), participants seeking care for post-acute cognitive complaints and a non-clinical group (*n* = 28), participants patients who did not seek care for post-acute COVID-19.	Significantly increased	Gupta et al., 2020b; Xin et al., 2021; Acosta-Ampudia et al., 2022; Ferrando et al., 2022; Hirzel et al., 2022; Lu et al., 2022; Schultheiss et al., 2022; Zhang et al., 2022b

Ischemia stroke (IS), Alzheimer’s disease (AD), Parkinson’s disease (PD), Amyotrophic lateral sclerosis (ALS), Multiple sclerosis (MS), Multiple system atrophy (MSA), mild cognitive impairment (MIC), Huntington’s Disease (HD), Lewy body dementia (LBD), Friedreich’s Ataxia (FA), beta-propeller protein-associated neurodegeneration (BPAN).

### Glial fibrillary acidic protein

Astrocytes are the most abundant cell type throughout the CNS and have many roles including but not limited to maintenance of BBB, neurotransmitter homeostasis, synaptogenesis, neurogenesis, ion and water homeostasis, and neuronal cholesterol synthesis (Cabezas et al., 2014; Liu et al., 2018). When neurological insult occurs, astrocytes become activated through reactive gliosis that involves the upregulation of glial fibrillary acidic protein (GFAP), a widely known biomarker of brain injury (Pekny and Pekna, 2014). As a structural protein that is unique to astrocytes, GFAP provides stability to astrocytes, thereby influencing their shape and movement (Eng et al., 2000; Hol and Capetanaki, 2017). Therefore, GFAP has been regarded as a biomarker of reactive astrocytes in a variety of neuropathological conditions (Eng et al., 2000). Elevated circulating levels of GFAP have been linked to a number of such neurological conditions including traumatic brain injury (TBI), spinal cord injury, multiple sclerosis (MS), Alzheimer’s Disease (AD), Alexander disease, Parkinson’s disease (PD), and neuromyelitis optica spectrum disorder (Elahi et al., 2020; Abdelhak et al., 2022; Heimfarth et al., 2022; Kim et al., 2022; Newcombe et al., 2022). It is evident that GFAP has been and continues to be explored as a potential biomarker of neurological injury across several neurodegenerative and inflammatory CNS diseases.

Recent studies have found elevated levels of GFAP in serum and/or plasma of COVID-19 patients (Kanberg et al., 2020, 2021; Frontera et al., 2022; Hanson et al., 2022; Sahin et al., 2022). This supports that GFAP correlates with disease severity, as it was found at significantly higher levels in COVID-19 patients who died during hospitalization when compared to those who survived (Frontera et al., 2022). Other results have supported elevated GFAP levels with disease severity but did not find a significant correlation with the presence of neurological symptoms (Sahin et al., 2022). One study found that GFAP levels normalized in all COVID-19 patients despite disease severity and the persistence of reported cognitive symptoms suggesting that the symptoms of COVID-19-associated cognitive impairment linger without the presence of active CNS injury (Kanberg et al., 2021). These findings may also further support the proposed mechanism that reactive gliosis following SARS-CoV-2 infection causes COVID-19-associated cognitive dysfunction by spreading hematogenously, infecting endothelial cells, and disrupting the BBB (Johansson et al., 2021; Mohamed et al., 2022). Taken together, these findings suggest that additional studies with larger sample sizes and standardized protocols should be explored to determine exactly how useful plasma or serum GFAP can be as a biomarker for COVID-19-associated cognitive impairment.

### Neurofilament light chain

Neurofilaments (Nfs) are classified as type IV intermediate filaments that provide cytoskeletal stability and allow for radial growth of neurons (Yuan et al., 2017; Gaetani et al., 2019). Under normal conditions, axons release neurofilament light chain (NfL), the most abundant subunit of Nfs, into the blood at low levels, and this has been found to increase with age (Yuan et al., 2017; Gaetani et al., 2019; Zanella et al., 2022). Moreover, during neurological degeneration or injury, these levels increase significantly indicating its potential use as a biomarker of neuroaxonal injury (Zanella et al., 2022). Elevated levels of NfL in serum have been associated with various neuropathologies such as cognitive decline, TBI, AD, PD, MS, Lewy body dementia (LBD), frontotemporal dementia (FTD), Amyotrophic Lateral Sclerosis (ALS), and Huntington Disease (HD) (Palermo et al., 2020; Rajan et al., 2020; Verde et al., 2021; Chouliaras et al., 2022; Ebenau et al., 2022; Newcombe et al., 2022; Thijssen et al., 2022).

Studies examining various COVID-19 patient populations have also found elevated plasma and or serum levels of NfL (Ameres et al., 2020; Kanberg et al., 2020, 2021; Aamodt et al., 2021; De Lorenzo et al., 2021; Prudencio et al., 2021; Frontera et al., 2022; Hanson et al., 2022; Verde et al., 2022). Similarly to GFAP, NfL was elevated in hospitalized patients who had COVID-19 encephalopathy (Hanson et al., 2022). NfL also correlates with disease severity as elevated plasma levels were found in COVID-19 patients that died during hospitalization (Aamodt et al., 2021; Frontera et al., 2022). When compared to the control group consisting of non-COVID-19 AD patients, the COVID-19 patients exhibited higher levels of NfL (Frontera et al., 2022). COVID-19 patients who did not have obvious signs or symptoms of cognitive dysfunction also had elevated levels of serum NfL (Prudencio et al., 2021; Verde et al., 2022). In another group of intensive care unit (ICU) COVID-19 patients, those who did not survive the infection had higher levels of NfL when compared to those who survived (Aamodt et al., 2021). Report shows that after 30-70 days, plasma NfL levels increased persistently and then normalized after six months in COVID-19 patients who continued to report the presence of neurological symptoms (Kanberg et al., 2021). Also plasma NfL levels were found to be increased from the first follow-up to the last in the severe group (Kanberg et al., 2020). Both studies support their shared hypothesis of delayed axonal injury occurring in severe COVID-19 patients, while astrocyte activation occurs earlier and is not limited to the severe COVID-19 patient population (Kanberg et al., 2020, 2021). The elevated concentrations of plasma NfL found in these COVID-19 patient populations warrants further investigation to explore its neuropathological mechanism causing neuroaxonal injury to determine whether it can be a contributing factor to the cognitive sequelae that arises in post-COVID-19 infections.

### Phosphorylated tau at threonine-181

The soluble tau proteins are important for maintaining neuronal microtubule integrity by providing stability and encouraging assembly (Wang and Mandelkow, 2016). The post-translational phosphorylation of tau is necessary for the protein to change its confirmation to operate under physiological conditions (Wang and Mandelkow, 2016; Kent et al., 2020). However, when phosphorylated excessively, the tau proteins dissociate from microtubules and aggregate with one another becoming insoluble and ultimately leading to extensive networks of neurofibrillary tangles (NFTs), which are characteristic of AD pathology (Metaxas and Kempf, 2016). The neurogenerative diseases distinctively express the hyperphosphorylation of Tau and subsequent aggregation are altogether known as tauopathies (Wang and Mandelkow, 2016). The role of p-tau 181 has been explored extensively in AD pathology and has been found to predict cognitive decline and AD several years before diagnosis and/or death (Guo et al., 2017; Lantero Rodriguez et al., 2020; Moscoso et al., 2021; Smirnov et al., 2022). These findings support p-tau 181 as a promising blood biomarker for AD and the potential for its application in other tauopathies.

Elevated levels of serum and/or plasma p-tau 181 have been found in COVID-19 patients (Sun et al., 2021; Frontera et al., 2022). COVID-19 patients who did not survive the infection and those who developed COVID-encephalopathy had elevated levels of p-tau 181, along with NfL and GFAP as mentioned previously. The study also found that hospitalized COVID-19 patients who experienced new cognitively related symptoms also had elevated levels p-tau 181 when compared to patients who did not experience additional cognitive sequelae (Frontera et al., 2022). In a study that examined the contents of neuronal-enriched extracellular vesicles (nEVs) in the plasma of COVID-19 patients, elevated levels of p-tau 181 were found and these levels also had a significant correlation with NfL in patients who reported neurological sequelae (Sun et al., 2021). There is some evidence suggesting that COVID-19 worsens pathology that has been implicated in AD such as tau, β-amyloid aggregation, neuroinflammation cerebral ischemia, and disruption of the BBB (Miners et al., 2020; Shen et al., 2022). Therefore, these findings suggest that p-tau 181 is yet another neurodegenerative biomarker correlated with COVID-19 disease severity during and/or following SARS-CoV-2 infection.

### Ubiquitin Carboxy-Terminal Hydrolase L1

Ubiquitin is a regulatory protein that is widely known for its role in the ubiquitin-proteasome system (UPS), which is involved in cellular processes including protein degradation, DNA repair and cell trafficking (Bishop et al., 2016; Guo and Tadi, 2022). In neurons, ubiquitination is involved in regulating the function of various synapses influencing their maintenance, transmission, and plasticity by altering the quantity of proteins at each synapse (Mabb and Ehlers, 2010). Deubiquinating enzymes known as deubiquitinases (DUBs) are responsible for removing ubiquitin from their target proteins (Bishop et al., 2016). Ubiquitin C-terminal hydrolase L1 (UCH-L1) is a specific member of this group that is highly expressed in neurons (Bishop et al., 2016). Higher levels of plasma UCH-L1 have been associated with PD (Ng et al., 2020), AD (Bogdan et al., 2022), Friedreich’s Ataxia (Zeitlberger et al., 2018), TBI (Wang et al., 2018), and general cognitive capabilities (Zhang et al., 2022a). The loss of UCH-L1 has resulted in the loss of neurons and instability of axons, while in some cases oxidatively modified UCH-L1 may aggregate (Bishop et al., 2016). These findings support that UCH-L1 is utilized as a general marker of neurodegeneration and other CNS-related complications.

Various COVID-19 patient populations have also experienced elevated levels of plasma UCH-L1 (Cooper et al., 2020; Frontera et al., 2022). It was found to correlate with COVID-19 disease severity as it was significantly higher in COVID-19 patients with encephalopathy (Frontera et al., 2022). As mentioned previously, hospitalized COVID-19 patients who experienced new neurological symptoms during admission had elevated plasma levels of UCH-L1, p-tau 181, and NfL, when compared to the control group consisting of non-COVID AD patients (Frontera et al., 2022). A group of ICU COVID-19 patients were also found to have higher levels of UCH-L1 that was also associated with delirium (Cooper et al., 2020). In another group of COVID-19 patients, UCH-L1 and NfL yielded predictive values on whether patients required a transfer to the ICU (De Lorenzo et al., 2021). Hence, it remains a possibility that UCH-L1 may be used as a prognostic biomarker when combined with others in providing potential clinical outcomes in COVID-19 patients (De Lorenzo et al., 2021).

### S100 calcium-binding protein B

The S100 protein family consists of proteins that principally bind Ca^2+^ and are named S100 because they dissolve in a neutral pH solution consisting of 100% saturated ammonium sulfate (Sedaghat and Notopoulos, 2008). A frequently investigated member of this protein family, S100 calcium-binding protein B (S100B), is used to describe levels of both the heterodimer S100AB and homodimer S100BB (Thelin et al., 2017). Serum levels of S100B may indicate astrocyte damage or injury, though with less accuracy than GFAP due to its more extensive distribution throughout different cell types of the CNS (Steiner et al., 2007). The function of S100B also differs depending on the concentration, having cytotoxic effects when increased (micromolar) and neuroprotective effects when at lower levels (nanomolar) in serum (Lam et al., 2013). S100B has been implicated in several neurological disorders including TBI (Thelin et al., 2017; Mondello et al., 2021), AD (Cristovao and Gomes, 2019), PD (Angelopoulou et al., 2021), ALS (Serrano et al., 2017), and MS (Barateiro et al., 2016). Micromolar levels of S100B is reported to cause such disorders by activating astrocytes and microglia, inducing nitric oxide (NO) release, increasing reactive oxygen species (ROS) and ultimately leading to neuroinflammation and loss of neurons (Michetti et al., 2019). These findings support that S100B is continuing to be explored as a potential blood biomarker across neurological disorders.

Elevated levels of circulating S100B has also been found in different groups of COVID-19 patients (Aceti et al., 2020; Mete et al., 2021; Savarraj et al., 2021; Sahin et al., 2022). As mentioned with previous brain injury biomarkers, serum S100B has also been associated with disease severity in COVID-19 patients (Aceti et al., 2020; Mete et al., 2021). Report show that levels of serum S100B were not correlated with neurological symptoms overall in acute phase COVID-19 patients, but did find marginally elevated levels of S100B in patients with more than one neurological symptom (Sahin et al., 2022). This may suggest that the elevated levels of S100B represents CNS injury to some extent during the acute phase of COVID-19, but it is unclear what implications this may have both clinically and in long-COVID patients. S100B has also been described as a pro-inflammatory ligand by binding to the Receptor for Advanced Glycation Endproducts (RAGE), which itself has been associated with neuroinflammation following neurological insult (Michetti et al., 2019). These findings may partly explain the association of elevated levels S100B with both disease severity and cognitive sequelae in COVID-19 infection. The exact role of S100B in COVID-associated cognitive dysfunction remains to be discovered to confirm whether it is directly contributing to neuropathological damage and/or it is a reaction of downstream inflammatory processes.

### Neuron specific enolase

Neuron specific enolase (NSE) is the gamma isozyme named due to its specificity for neuronal and neuroendocrine cells (Haque et al., 2018). NSE itself can be expressed as two different isozymes in neurons as either γγ or αγ (Polcyn et al., 2017). In astrocytes, NSE is expressed as γγ and in oligodendrocytes and microglia it is found as the αγ subunits (Polcyn et al., 2017). NSE has therefore been linked to both neurological and non-neurological pathologies due to its tissue specificity and upregulation following axonal injury (Polcyn et al., 2017). Similar to S100B, NSE can be both neuroprotective or neuroinflammatory depending on surrounding conditions such as the typical homeostatic environment, disease state, or presence of injury (Polcyn et al., 2017). The neuropathological conditions that have been associated with altered levels of plasma or serum NSE include AD (Chaves et al., 2010), HD (Ciancarelli et al., 2014), postoperative cognitive dysfunction (POCD) (Wan et al., 2021), and beta-propeller protein-associated neurodegeneration (BPAN) (Takano et al., 2017).

Neuron specific enolase levels have also been found at higher concentrations in the serum or plasma of COVID-19 patients (Wei et al., 2020; Cione et al., 2021; Savarraj et al., 2021). Increased levels of serum NSE has also been associated with disease severity as mentioned previously with other biomarkers specifically in a cohort of COVID-19 patients who developed dyspnea (Cione et al., 2021), in critical cases of COVID-19 patients (Wei et al., 2020), and in patients immediately following hospital admission for COVID-19 infection (Savarraj et al., 2021). A unique observation found was that serum NSE was found at significantly higher levels in men when compared to women, which may support increased susceptibility to COVID-associated cognitive dysfunction in men (Savarraj et al., 2021). NSE may be elevated in COVID-19 due to the potential presence of axonal injury (Polcyn et al., 2017), lung injury (Cione et al., 2021), neuroinflammation (Haque et al., 2018), or a combination of all. There is not enough data at this time to concretely validate the use of serum NSE as a biomarker of only neurodegeneration and/or prognosis in COVID-19 infection. Further investigation are required to support these findings and uncover the exact role of NSE in COVID-29 infection.

### Inflammatory cytokines

Pro-inflammatory cytokines, such as interleukin (IL)-6, IL-1β, and tumor necrosis factor-α (TNF-α) are well established as major contributing factors to neuropathological diseases (Wang et al., 2015; Gupta et al., 2020b; Xin et al., 2021; Lu et al., 2022). Anti-inflammatory cytokines such as IL-10 also play crucial roles in brain injury and neuroinflammation due to its ability to suppress inflammatory responses (Garcia et al., 2017; Burmeister and Marriott, 2018; Lu et al., 2022; Sanchez-Molina et al., 2022). C-reactive protein (CRP), a non-specific marker of systemic inflammation, is induced by pro-inflammatory cytokines such as IL-6, and has been associated with chronic inflammation, and various degrees of cognitive dysfunction (Watanabe et al., 2016; Luan and Yao, 2018; Vintimilla et al., 2019; Gupta et al., 2020b; Xin et al., 2021). A cascade of events, referred to as “cytokine storm” or “cytokine release syndrome (CRS),” has been implicated in neurotoxicity, disruption of the integrity of BBB, neuroglial cells activation, and ultimately neuroinflammation (Gupta et al., 2020b; Zhang et al., 2022b).

In COVID-19 patients, elevated serum levels of IL-6, IL-1β, TNF- α, IL-10, and CRP have been measured and discussed (Chen et al., 2020; Han et al., 2020; Islam et al., 2021a; Lavillegrand et al., 2021; Lu et al., 2021; Acosta-Ampudia et al., 2022; Ferrando et al., 2022; Hirzel et al., 2022; Leretter et al., 2022; Montazersaheb et al., 2022; Peluso et al., 2022; PHOSP-COVID Collaborative Group, 2022; Schultheiss et al., 2022). IL-6, CRP, and IL-10 and have also been associated with disease severity amongst COVID-19 patients, correlating with severe clinical outcomes and fatality (Han et al., 2020; Lavillegrand et al., 2021; Alshammary et al., 2022; Ashktorab et al., 2022; Azaiz et al., 2022; Galliera et al., 2022; Jafrin et al., 2022; Mainous et al., 2022). CRP was found specifically to be positively correlated with two parts of a Continuous Performance Test (CPT) conducted in patients who had resolved COVID-19 infections (Zhou et al., 2020a) and was found at significantly elevated concentration in COVID-19 patients with moderate to severe cognitive dysfunction (Arica-Polat et al., 2022). Even though vast amount of evidence continues to validate the role of hyperinflammation in SARS-CoV-2 infection, there is a clear need for additional studies to explore the role of these inflammation in the CNS in COVID-19 patient populations.

## Role of circulating micro RNAs in COVID-19-associated cognitive dysfunction

Growing evidence suggests that as post-transcriptional regulators of gene expression, miRNAs are involved in physiological and pathological processes and their dysregulation in function is synonymous with a multiplicity of diseases (Condrat et al., 2020; Carini et al., 2021). The prominent role of non-coding microRNAs in CNS and their signature in the circulation has been well established in various neurodegenerative diseases (Thounaojam et al., 2013; Bahlakeh et al., 2021; Islam et al., 2021c; Perdoncin et al., 2021; Blount et al., 2022). Hence, miRNAs as possible therapeutic targets and disease markers for early diagnosis have strongly been advocated because of their stability and convenience in extraction from biological fluids (Szelenberger et al., 2019). In this section of the review, we are showcasing the importance of some dysregulated miRNAs in COVID-19 and their possible correlation with CNS to further explore the mechanism of COVID-19- associated cognitive dysfunction. A summary of the findings are illustrated in Table 2.

**TABLE 2:** Summary of circulating miRNAs associated with neurological dysfunction showing potential dysregulation in COVID-19.

miRNA	Source	Target genes	Status in neurodegenerative diseases	Patients’ information	Status in COVID-19	References
miR-146a	Serum	IRAK1, TRAF6	IS-decreased AD-decreased PD-decreased	1.Different grades of COVID-19 patients (n = 103) 2. 13 COVID-19 patients, characterized by multifocal interstitial pneumonia confirmed by CT-scan and requiring oxygen therapy.	Significantly decreased	Fan et al., 2020; Nakano et al., 2020a,b; Keikha and Jebali, 2021; Keikha et al., 2021; Sabbatinelli et al., 2021
miR-155	Serum	SOCS1, SHIP1, STAT5, IL13Ra1, claudin-1, annexin-2, syntenin-1, DOCK-1	IS-increased AD-increased PD-increased ALS-increased MS-increased	1. 18 patients after diagnosis of Covid-19 and in the recovery period. 2. 20 patients with COVID-19 infection in the acute period and in the recovery period. 3. 150 COVID-19 patients classified into two main groups: moderate patients and severe patients.	Significantly increased	Lopez-Ramirez et al., 2014; Song and Lee, 2015; Donyavi et al., 2021; Zingale et al., 2021; Abbasi-Kolli et al., 2022; Haroun et al., 2022
Let-7b	PBMC	TLR7, HMGA2	AD-increased PD-increased MIC-increased	1. 18 patients after diagnosis of COVID-19 and in the recovery period. 2. 31 COVID-19 positive obese female participants.	Significantly increased	Coleman et al., 2017; Donyavi et al., 2021; Huang et al., 2021b; Qin et al., 2021; Bellae Papannarao et al., 2022
miR-31	Serum	RhoA, APP, BACE1, PARK2, GIGYF2	AD-decreased PD-decreased MSA-decreased	1.Different grades of COVID-19 patients (n = 103) 2. 122 COVID-19 patients with different severity of illness. 3. 10 COVID-19 patients 2–15 days (average 8 days) post symptomatic disease onset.	Significantly decreased	Pearn et al., 2018; Barros-Viegas et al., 2020; Li et al., 2020; Tang et al., 2020; Yan et al., 2020; Bautista-Becerril et al., 2021; Farr et al., 2021; Keikha and Jebali, 2021; Keikha et al., 2021
miR-16	Plasma	APP, BACE1, Tau	AD-decreased	1. 84 COVID-19 patients divided according to the severity of the disease. 2. 94 COVID-19 patients	Significantly decreased	Liu et al., 2012; Parsi et al., 2015; De Gonzalo-Calvo et al., 2021; Li et al., 2022b
miR-21	Plasma/serum	NF-κB, PTEN/AKT,PI3K, GSK-3β, mTOR1, STAT3	AD-decreased PD-decreased IS-decreased	1. 10 COVID-19 patients 2. 13 COVID-19 patients, characterized by multifocal interstitial pneumonia confirmed by CT-scan and requiring oxygen therapy 3. 122 COVID-19 patients with different severity of illness. 4. 6 severe and 6 moderate COVID-19 patients	Significantly decreased	Ma et al., 2011; Feng et al., 2018; Gao et al., 2020; Bai and Bian, 2022; Blount et al., 2022

Ischemia stroke (IS), Alzheimer’s disease (AD), Parkinson’s disease (PD), Amyotrophic lateral sclerosis (ALS), Multiple sclerosis (MS), Multiple system atrophy (MSA), mild cognitive impairment (MIC), Peripheral blood mononuclear cell (PBMC), interleukin-1 receptor-associated kinase 1 (IRAK1), receptor-associated factor 6 (TRAF6), Suppressor of Cytokine Signaling 1 (SOCS1), SH2 Domain-Containing Inositol 5’-Phosphatase1 (SHIP1), Signal Transducers and Activators of Transcription 5 (STAT5) and IL-13 Receptor Alpha 1 (IL13Ra1), Dedicator of cytokinesis 1 (DOCK-1), toll-like receptor 7 (TLR7), High-mobility group AT-hook 2 (HMGA2), amyloid precursor protein (APP), β-secretase (BACE1), parkin E3 ubiquitin-protein ligase (PARK2), interacting GYF protein 2 (GIGYF2), Ras Homolog Family Member A (RhoA), tubulin associated unit protein (TAU protein), Nuclear factor kappaβ (NF-κβ), Phosphatase and tensin homolog (PTEN), Phosphoinositide 3-kinase (PI3K), Mammalian target of rapamycin complex 1 (mTOR1), Glycogen Synthase Kinase 3 Beta (GSK-3β), toll-like receptor 4 (TLR4).

### miR-146a

miR-146a is produced by bone marrow mesenchymal stem cells and released in exosome granules, then it is taken up by activated astrocytes, particularly in the hippocampal region, indicating it may serve a neuroprotective role in seizure-related cognitive dysfunction (Kong et al., 2015). miR-146a exerts an anti-inflammatory effect by inactivating NF-κB activity through a reduction of interleukin-1 receptor-associated kinase 1 (IRAK1) and tumor necrosis factor associated factor 6 (TRAF6) (Nakano et al., 2020a,b). This will further lead to the supression of NF-κB’s target genes such as the interleukins IL-6, IL-8, IL-1β, and TNF alpha (TNF-α) (Saba et al., 2014; Fan et al., 2020). Increased expression of miR-146a in brain endothelial cells alters cytokine signaling and reduces NF-κB activity by reducing its nuclear translocation and thus decreasing the number of expressed T-cell adhesion molecules and limiting their entry into the CNS in the development of neuroinflammation (Wu et al., 2015). Circulating miR-146a is reduced in the blood of AD (Kumar and Reddy, 2016; Swarbrick et al., 2019), reducing the capability to deal with neurodegenerative inflammation. Overexpression of miR146a in microglia has been shown to reduce cognitive deficits in learning and memory, attenuate neuroinflammation, reduce beta-amyloid levels, and alleviate plaque-associated neuritic pathologies. miR-146a also influences microglial phenotype switching, allowing for the reduction of pro-inflammatory cytokine production and improved phagocytic functions in the clearance of beta-amyloid and tau (Liang et al., 2021). Thus, serum miR-146a levels are being considered for clinical use as a biomarker for neurodegenerative diseases (Kumar and Reddy, 2016; Mai et al., 2019; Swarbrick et al., 2019; Sabbatinelli et al., 2021).

Cumulative evidences suggest that decreased expression of miR-146a is associated with SARS-CoV-2 infection (Keikha and Jebali, 2021; Roganovic, 2021; Sabbatinelli et al., 2021). Furthermore, individuals with pre-existing inflammatory conditions which cause a decreased expression of miR-146a are thus predisposed to COVID-19 infection, and at risk for more serious progression of the illness (Roganovic, 2021; Sudhakar et al., 2022). Interestingly, COVID-19 patients showed a down-regulation of this anti-neuroinflammatory miRNA, which in turn causes an increase in expression of IL-6, IL-8, IL-17, and other inflammatory cytokines (Arghiani et al., 2021; Roganovic, 2021). Increased levels of the inflammatory cytokine IL-6 thus reduce the effectiveness of many drugs being currently tested for use against COVID, such as tocilizumab, because they act as antibodies against these inflammatory cytokines (Arghiani et al., 2021; Sabbatinelli et al., 2021). Conversely, some studies have shown that the expression of miR-146a is increased in COVID-19 patients when compared to healthy controls (Donyavi et al., 2021; Pinacchio et al., 2022). miR-146a is therefore uniquely can be positioned as one of a handful of micro-RNAs suited for use as a biomarker for cognitive dysfunction and SARS-CoV-2 infection and as a potential therapeutic for the treatment of those disease states. Given the altered expression of miR-146a in neurodegenerative diseases as well as in SARS-CoV-2 infection, and its role as an anti-neuroinflammatory microRNA, future studies with large populations may help to elucidate the actual mechanism of action of miR-146a in COVID-19 mediated cognitive decline and its importance as a circulating prognostic marker.

### miR-155

CNS upregulation of miR-155 has been associated cognitive dysfunction and is the most expressed chromosome 21 miRNA in Down’s Syndrome dementia, as it is co-expressed with hyperphosphorylated tau protein (Tili et al., 2018). miR-155 act as a prevalent CNS pro-inflammatory mediator and microglia activator by regulating inflammatory cytokines such as (IFN)-λ and IFN-β (Thounaojam et al., 2013). In the CNS, the action of miR-155 is mediated in microglia and macrophages through NF-κB following stimulation of the appropriate TLR and interferon-gamma release. It also causes a reduction in the anti-inflammatory response by targeting anti-inflammatory regulators such as Suppressor of Cytokine Signaling 1 (SOCS1), SH2 Domain-Containing Inositol 5’-Phosphatase1 (SHIP1), activator protein 1, Signal Transducers and Activators of Transcription 5 (STAT5) and IL-13 Receptor Alpha 1 (IL13Ra1), further increasing inflammation (Song and Lee, 2015; Zingale et al., 2021). miR-155 increases BBB permeability by targeting cell–cell complex molecules including claudin-1 and annexin-2 and focal adhesion components such as syntenin-1 and dedicator of cytokinesis 1 (DOCK-1) (Lopez-Ramirez et al., 2014). miR-155 is also associated with promotion of CNS T cell responses and the subsequent development of cognitive dysfunction symptomology. Through regulation of interferon-gamma signaling, miR-155 can influence CD8 + T cell activation, T cell development, various cell to cell interactions, and macrophage activation. T cell activation and IFN-y production, followed by infiltration into the CNS, results in the deposition of beta-amyloid and thus cognitive dysfunction (Song and Lee, 2015). The pro-neuroinflammatory role of miR-155 was affirmed through knockout studies which show reduced neuroinflammation, reduced cognitive impairment and better recovery in traumatic brain injury mouse models (Henry et al., 2019). Moreover, miR-155 overexpression is implicated in CCR2/CXCL2 translation disorders, causing impaired cell migration and clearance of beta-amyloid by blood-derived monocytes (BDMs) and monocyte-derived macrophages (MDMs) in AD (Guedes et al., 2016). The pro-inflammatory function of miR-155 also carries over into auto-immune conditions such as MS-associated cognitive dysfunction by promoting inflammatory damage to the neurovascular units of the blood-brain-barrier *via* down regulation of junctional proteins (Maciak et al., 2021). miR-155 contributes to CNS demyelination *via* microglia activation and subsequent production of TNF-a, IL-1, IL-6, interferon-inducible protein 10 (IP-10), macrophage inflammatory protein-1a (MIP-1a), monocyte chemoattractant protein-1 (MCP-1), and nitric oxide (NO) (Miller, 2012). It is reported that miR-155 mediated impairment to the BBB, damage of myelin and axons, synaptic dysfunction, and dysregulated neurotransmitter production due to acute inflammation can lead to brain atrophy and progressive cognitive impairment (Varma-Doyle et al., 2021).

Serum miR-155 levels are significantly increased during the acute and post-acute phases of SARS-CoV-2 infection (Bautista-Becerril et al., 2021; Abbasi-Kolli et al., 2022). The study which showed significantly increased expression of miR-155 in the peripheral blood mononuclear cell (PBMC) samples of patients with acute COVID-19 infection suggest it as a diagnostic marker for COVID-19 (Abbasi-Kolli et al., 2022). Similarly, another study demonstrates miR-155 as a biomarker to distinguish acute from post-acute phase of COVID-19 disease (Donyavi et al., 2021). Additionally, plasma miR-155 levels appear to be significantly correlated with chest CT findings, CRP and ferritin levels, mortality, d-dimer, WBC count and neutrophil percentage. miR-155 levels are 90% sensitive and 100% specific when used as a biomarker for the detection of COVID-19 and are 76% sensitive and specific for detection of severity of COVID-19 disease (Haroun et al., 2022). Overexpression of miR-155 in SARS-CoV-2 infection thus may partially explain the enhanced immune response that leads to CNS damage in the context of covid-associated cognitive dysfunction.

### Let-7b

Let-7b a multifunctional miRNA that is differentially expressed in issues of cognitive dysfunction in comparison to healthy individuals (Rahman et al., 2020; Yuen et al., 2021). Levels of Let-7b appear to be increased in diseases of cognitive dysfunction such as MCI (Kenny et al., 2019), AD (Leidinger et al., 2013), and PD (Huang et al., 2021b). Overexpression of Let-7b in AD models was found to significantly reduce cell viability, inhibit autophagy and increase apoptosis through increased cleavage of caspase 3 and through increased expression levels of PI3K, p-AKT, and p-mTOR in upstream signaling pathways (Pang et al., 2022). Let-7b also appears to be involved in neurodegeneration through interaction with toll-like receptor 7 (TLR7) (Lehmann et al., 2012). TLR7 mediated pathway of Let-7b action is additionally seen in the postmortem hippocampal formations of alcoholics, where TLR7 and Let-7b expression was increased, leading to neuroinflammation and neurodegeneration (Coleman et al., 2017). Additional studies have also shown the role of Let-7b and TLR7 mediated mechanism of alcohol-associated cognitive dysfunction (Qin et al., 2021). Let-7b has been shown to regulate the function of high mobility group AT-hook 2 (HMGA2) protein in PD, causing a dysregulation of chromatin structure and transcription which leads to decreased self-renewal of neuronal stem cells, leading to neurodegeneration (Huang et al., 2021b).

Let-7b levels are elevated in peripheral blood samples in both the acute and post-acute stages of SARS-CoV-2 infection compared to healthy individuals (Donyavi et al., 2021; Nain et al., 2021), suggesting potential use as a clinical biomarker COVID-19 infection. Let-7b targets ACE2 causing dysregulation of ACE2 and potentially increasing susceptibility to SARS-CoV-2 infection, making it a potential target for therapeutic treatment of SARS-CoV-2 infection (Bellae Papannarao et al., 2022). Let-7b, in the context of SARS-CoV-2 infection, increases apoptosis through a reduction of BCL-2, an anti-apoptotic protein, and through modulation of immune responses, establishing a potential link between chronic inflammatory illness such as type 2 diabetes and COVID-19 (Islam et al., 2021b), which may have effect on cognitive dysfunction. Reports shows showcase Let-7b as a marker of lung disease which is highly prevalent in COVID-19 (Islam et al., 2021b; Nain et al., 2021). These reported upregulation of Let-7b in SARS-CoV-2 infection suggest its possible link with cognitive dysfunction that warrants future studies.

### miR-31

miR-31 is decreased in the serum of AD individuals compared to healthy controls (Dong et al., 2015; Klyucherev et al., 2022) and can be used as part of a panel in conjunction with miR-93 and miR-146a to differentiate Alzheimer’s Disease from Vascular Dementia (Dong et al., 2015). Expression of miR-31 was also decreased in the serum of PD and Multiple System Atrophy (MSA) individuals (Yan et al., 2020). Letiviral delivery of miR-31 was able to significantly ameliorate AD neuropathology by reducing Aβ deposition in both the hippocampus and subiculum of transgenic mice models (Barros-Viegas et al., 2020). The study shows that miRNA-31 targets amyloid precursor protein (APP) and β-secretase (BACE1), which further abolishes the pathogical aletrations in AD. The results showed improvements in memory deficits, reduced anxiety, and reduced cognitive inflexibility, suggesting future possibilities for miR-31 to be used as a therapeutic in the treatment of AD (Barros-Viegas et al., 2020). RhoA has been reported to modulate synaptic plasticity and inhibition of the RhoA pathway reduces cognitive impairment and deficits in synapses and dendritic spines (Pearn et al., 2018). miR-31 has been reported as a regulator of RhoA and decrease in miR-31 plays a role in the development of cognitive dysfunction in learning, memory, behavior, etc., patterns which are similarly seen in neurodegenerative disease (Qian et al., 2021). miRNA target prediction analysis have shown some PD- and MSA-related genes such as parkin E3 ubiquitin-protein ligase (PARK2), GRB10-interacting GYF protein 2 (GIGYF2) as potential target of miR-31 (Yan et al., 2020).

miR-31 is multifunctional in the context of COVID-19, particularly when discussing hypoxia and potential resultant neurodegenerative effects. miR-31 serum expression levels have been demonstrated to be decreased in COVID-19 infected patients (Bautista-Becerril et al., 2021). Expression levels of miR-31 appear to decrease with worsening severity of illness with COVID-19 infection also, making it a worthwhile candidate for use as a biomarker of COVID-19 infection and severity (Keikha et al., 2021). Decreased expression may play a role in the neurodegenerative pathologies seen with enhanced micro coagulation in SARS-CoV-2 infected individuals. Thus, decreased levels of miR-31 appear to have a multifactorial effect in cognitive dysfunction and in SARS-CoV-2 infection and presents as a potential link between the two disease processes. Conversely, microRNA expression profile analysis of another set of COVID-19 patients showed up-regulation of miR-31 expression (Farr et al., 2021). Hence, future studies with more population size and more detailed mechanistic approach may clarify the exact role of miR-31 in COVID-19-associated cognitive decline.

### miR-16

miR-16 is differentially expressed in various neurodegenerative diseases, with its levels being significantly decreased in the serum of AD patients (Denk et al., 2018; Mckeever et al., 2018). miR-16 regulates cell death in AD by targeting APP (Liu et al., 2012; Zhang et al., 2015; Turk et al., 2021). Downregulation of miR-16 in hippocampal neurons has been associated with increases in APP eventual processing to beta-amyloid followed by deposition into neurons within the brain (Zhang et al., 2015; Grinan-Ferre et al., 2018). In cell culture studies, miR16 has been shown to regulate Aβ production, and Tau phosphorylation (Hebert et al., 2012). Similarly report shows a reduction of the expression of a number of genes related to AD including APP, BACE1, tau, inflammation and oxidative stress through the delivery of miR-16 mimics directly to mouse brain (Parsi et al., 2015). The role of miR16 in targeting genes involved in neurite extension and branching in hippocampal neurons during presymptomatic prion disease has also been reported (Burak et al., 2018). miR-16 appears to have potential for future drug development because it simultaneously targets various endogenous targets of AD biomarkers. These findings suggest that further research is needed into the role of miR-16 in other forms of neurodegenerative diseases to evaluate its impact more completely on cognitive function.

Serum miR-16 levels are likewise reduced in COVID-19 infected patients suggesting a potential link between differential miR-16 expression and covid-associated cognitive dysfunction. miR-16 levels were established to be inversely correlated with length of ICU stay in COVID-19 infected patients as well, opening the possibility for its use as a biomarker of disease and severity (De Gonzalo-Calvo et al., 2021). Also, miR-16 has already been used as a biomarker for other viral respiratory illnesses such as community acquired pneumonia (Galvan-Roman et al., 2020). miR-16 is capable of high affinity binding to the SARS-CoV-2 genome, opening future avenues of potential drug research (Kim et al., 2020; Nersisyan et al., 2020). A single-cell RNA-sequencing based study identified miR-16 as a potential virus targeting miRNAs across multiple cell types from bronchoalveolar lavage fuid samples (Li et al., 2022b). Down regulation of miR-16 levels in individuals with SARS-CoV-2 suggests miR-16 may play a role in covid-associated cognitive dysfunction due to its previously defined role in other forms of neurodegenerative cognitive dysfunction.

### miR-21

miR-21 is extensively involved in processes governing apoptosis and neuroinflammation in neurodegenerative diseases and thus in cognitive dysfunction (Bai and Bian, 2022). Serum and CSF levels of miR-21 are decreased in patients with AD compared to individuals with Lewy Body Dementia and healthy controls (Gamez-Valero et al., 2019). miR-21 acts as an anti-inflammatory microRNA by acting as a negative feedback regulator on NF-κB in response to pro-inflammatory signaling (Ma et al., 2011). miR-21 has been shown to ameliorate cognitive impairments associated with brain injury from subarachnoid hemorrhaging by modulation of the PTEN/AKT pathway and reducing apoptosis in the hippocampus and prefrontal cortex (Gao et al., 2020). Use of miR-21 mimics in cell culture studies of AD has shown that miR21 is capable of inhibiting beta-amyloid induced apoptosis by increasing expression of PI3K, AKT, and GSK-3B (Feng et al., 2018). Overexpression of miR-21 was demonstrated to protect neurons of the hippocampus in epileptic rat studies by inhibiting STAT3 (Bai and Bian, 2022). Microglial miR-21 has been reported to protect neurons from cell death under hypoxic conditions (Zhang et al., 2012). miR-21 has been shown to restore neurogenesis and reverse cellular senescence *via* inhibition of the mTOR1 pathway in models of vascular dementia, making a candidate as a potential therapeutic in the treatment of vascular dementia and its associated cognitive impairment (Blount et al., 2022).

Serum miR-21 levels have been reported to be decreased in COVID-19 infected individuals (Li et al., 2020; Sabbatinelli et al., 2021). The down-regulation in the relative expression of miR-21 in COVID-19 patients was concomitant with up-regulation of its target proinflammatory genes (Keikha and Jebali, 2021). The study also demonstrate miR-21 as an anti- neuroinflammatory miRNA, for correlating the disease grade from asymptomatic to critical illness in COVID-19. Down regulation of miR-21 in COVID-19 patients exacerbates systemic inflammation through hyperactive immune response, loss of T cell function, and immune dysregulation (Tang et al., 2020). Increased systemic inflammation can weaken the blood-brain-barrier, causing heightened neuroinflammation and resulting in neurodegeneration. Thus, decreases in expression of miR-21 could directly and indirectly contribute to the development and progression of covid-associated cognitive dysfunction, or worsening of pre-existing cognitive dysfunction after infection with SARS-CoV-2.

## Conclusion

The different sequelae presented by post-COVID-19 patients are being increasingly studied from the improvement of clinical and laboratory experience. Cumulative evidences suggest that surviving patients of COVID-19 have a high risk of developing some neuropsychiatric impairment, which can occur in different forms, such as cases of depression, anxiety, and severe mental illness. The sequelae related to cognitive decline and neurodegeneration are diverse and there is a need for detailed assessments to identify new neurological conditions. An extremely relevant factor to be considered in the fight against COVID-19 is the use of biomarkers in the early recognition of patients susceptible to developing the severe form of the disease. The discovery of potential markers could be used to provide essential information that will assist in stratifying these patients, improving primary care, and developing optimal individualized therapy according to the patient’s response to cognitive damage. The review summarizes the neuropathological changes associated with COVID-19 and signifies the importance of circulating biomarkers and miRNAs in these neurodegenerative changes (Figure 3). Thus, the clinical use of the markers reported in this review will significantly improve the development of new policies to prevent, address and manage the neurological conditions caused by SARS-CoV-2 infection and may aid in future research exploring the mechanistic aspects of COVID-19 associated neurodegeneration and cognitive dysfunction.

**FIGURE 3:** Schematic representation of the main mechanisms involved in the neurophysiology caused by SARS-CoV2 virus and the role of biomarkers and miRNAs in neuronal damage. The SARS-CoV2 virus has the ability to infect brain tissue by mechanisms involving the olfactory and hematological pathway, which will lead to an oxidative and inflammatory state in nervous tissue, due to the activation of neutrophils, astrocytes, and microglial cells releasing excessive ROS and pro-inflammatory molecules. The imbalance in brain homeostasis leads to a dysfunction in the expression pattern of different biomarkers and miRNAs, potentiating neuroinflammatory mechanisms, responsible for brain damage and the consequent progression of cognitive dysfunction and neurodegenerative disorders. GFAP, Glial fibrillary acid protein; NFL, Neurofilament light chain; P-tau-181, Phosphorylated tau at threonine-181; UCH-L1, Ubiquitin Carboxy-Terminal Hydrolase L1; S100B, S100 calcium-binding protein B; NSE, Neuron Specific Enolase.

## Author contributions

SP: conceptualization, project administration, and writing—review and editing. KS: conceptualization and project administration. MA, ET, BG, DP, RP, and NF: writing—original draft preparation. All authors contributed to the article and approved the submitted version.
